This article has been retracted.

# Propylthiouracil prevents cutaneous and pulmonary fibrosis in the reactive oxygen species murine model of systemic sclerosis

**DOI:** 10.1186/ar4300

**Published:** 2013-09-16

**Authors:** Gianluca Bagnato, Alessandra Bitto, Natasha Irrera, Gabriele Pizzino, Donatella Sangari, Maurizio Cinquegrani, William Neal Roberts, Marco Atteritano, Domenica Altavilla, Francesco Squadrito, Gianfilippo Bagnato, Antonino Saitta

**Affiliations:** 1 Department of Clinical and Experimental Medicine, Division of Internal Medicine, University of Messina, Via Consolare Valeria n°1, 98100, Messina, Italy; 2 Department of Clinical and Experimental Medicine, Division of Pharmacology, University of Messina, Via Consolare Valeria n°1, 98100, Messina, Italy; 3 Department of Clinical and Experimental Medicine, Division of Rheumatology, University of Messina, Via Consolare Valeria n°1, 98100, Messina, Italy; 4 Department of Internal Medicine, Division of Rheumatology, University of Louisville, Louisville, KY 40292, Kentucky, USA

## Abstract

**Introduction:**

Recent advances suggest that the cellular redox state may play a significant role in the progression of fibrosis in systemic sclerosis (SSc). Another, and as yet poorly accounted for, feature of SSc is its overlap with thyroid abnormalities. Previous reports demonstrate that hypothyroidism reduces oxidant stress. The aim of this study was therefore to evaluate the effect of propylthiouracil (PTU), and of the hypothyroidism induced by it, on the development of cutaneous and pulmonary fibrosis in the oxidant stress murine model of SSc.

**Methods:**

Chronic oxidant stress SSc was induced in BALB/c mice by daily subcutaneous injections of hypochlorous acid (HOCl) for 6 weeks. Mice (*n *= 25) were randomized into three arms: HOCl (*n *= 10), HOCl plus PTU (*n *= 10) or vehicle alone (*n *= 5). PTU administration was initiated 30 minutes after HOCl subcutaneous injection and continued daily for 6 weeks. Skin and lung fibrosis were evaluated by histologic methods. Immunohistochemical staining for alpha-smooth muscle actin (α-SMA) in cutaneous and pulmonary tissues was performed to evaluate myofibroblast differentiation. Lung and skin concentrations of vascular endothelial growth factor (VEGF), extracellular signal-related kinase (ERK), rat sarcoma protein (Ras), Ras homolog gene family (Rho), and transforming growth factor (TGF) β were analyzed by Western blot.

**Results:**

Injections of HOCl induced cutaneous and lung fibrosis in BALB/c mice. PTU treatment prevented both dermal and pulmonary fibrosis. Myofibroblast differentiation was also inhibited by PTU in the skin and lung. The increase in cutaneous and pulmonary expression of VEGF, ERK, Ras, and Rho in mice treated with HOCl was significantly prevented in mice co-administered ////with PTU.

**Conclusions:**

PTU, probably through its direct effect on reactive oxygen species or indirectly through thyroid function inhibition, prevents the development of cutaneous and pulmonary fibrosis by blocking the activation of the Ras-ERK pathway in the oxidant-stress animal model of SSc.

## Introduction

Theories of scleroderma pathogenesis accommodate three fundamental and long-standing observations about systemic sclerosis (SSc): its vascular nature, its abnormal fibroblast activation, and the immune-mediated damage [1]. In spite of a significant effort, the etiopathogenesis of SSc remains unknown. A link between reactive oxygen species and pathogenesis of scleroderma has been explored [2]. Oxidative stress may directly or indirectly stimulate the accumulation of extracellular matrix proteins. Conversely, fibrosis may contribute to oxidative stress, or both of them may be triggered by an independent mechanism. Indirect proof of abnormal oxidative stress was provided by Dooley *et al*. [3], who showed that the antioxidant epigallocatechin-3-gallate can reduce extracellular matrix production and inhibit contraction of dermal fibroblasts from systemic sclerosis patients. Furthermore, epigallocatechin-3-gallate was able to suppress intracellular reactive oxygen species (ROS), extracellular signal-regulated kinases (ERK1-2) signaling, and nuclear factor kappa-light-chain-enhancer of activated B cells (NF-κB) activity [4]. ERK, one of the relevant targets of ROS, and its upstream mediators, such as Ras family proteins, function as key molecules in the pathway that leads to fibrosis, and in maintaining the generation and amplification of ROS. Levels of ROS and type I collagen were significantly higher, and amounts of free thiol were significantly lower in SSc fibroblasts compared with normal fibroblasts [5]. Hormonal influences on the etiopathogenesis of the disease have been intensively studied, focusing on disturbances of the gonadal axis [6,7]. A second, and as yet poorly accounted for, endocrine feature of scleroderma is its overlap with thyroid abnormalities [8]. Of 719 patients affected by SSc, 273 (38%) had at least one other autoimmune disease, with the most frequent being autoimmune thyroid disease (AITD) [9]. Whereas the association of Graves disease with SSc [10,11] is supported by case reports, the literature related to Hashimoto thyroiditis and hypothyroidism in general, either subclinical or symptomatic, in SSc patients is more robust [12]. It was recently demonstrated by Cianfarani *et al*. [13] that thyroid-stimulating hormone (TSH)-receptor messenger RNA is consistently detected in both skin biopsies and cultured primary keratinocytes and, more interestingly, in dermal fibroblasts of patients with SSc. A previous report confirmed the occurrence of a state of oxidizing stress in relation to hyperthyroidism [14].

The aim of the study was, therefore, to evaluate the effect of propylthiouracil (PTU), administered at a dose able to induce hypothyroidism, on the extent of fibrosis in a murine model of SSc, based on reactive oxygen species-mediated injury.

## Materials and methods

### Animals

Pathogen-free, 6-weeks-old female BALB/c mice were purchased from Harlan (///Italy), maintained with food and water *ad libitum*, and given human care according to institutional guidelines. The project was reviewed and approved by the Ethics Committee of the University of Messina. All mice were housed in single cages under controlled light and temperature conditions. Mice (*n *= 25) were randomized in three arms: HOCl alone (*n *= 10), HOCl plus propylthiouracil (*n *= 10; hereinafter PTU), or vehicle alone (*n *= 5; subsequently SHAM) for 6 weeks.

### ROS preparation and treatments

SSc was induced as characterized in detail in the Cochin chronic oxidant stress model [15]. In brief, hypochlorous acid (HOCl) was produced by adding 166 μl of sodium hypochlorite (NaClO) solution (2.6% as active chlorine) to 11.1 ml of potassium hydrogen phosphate (KH_2_PO_4_) solution (100 m*M*; pH 7.2). A total of 100 μl of solution containing HOCl was injected s.c. into the back of the mice, by using a 27-gauge needle, every day for 6 weeks. Mice (*n *= 10) from the HOCl group (*n *= 20) were randomly chosen to be treated with propylthiouracil (Sigma-Aldrich, Italy///) at the dose of 12 mg/kg/day. The dosage of 12 mg/kg/day was chosen as being consistent with the report from the European Medicines Agency recommendations on propylthiouracil, based on previously published studies. The method and PTU-dosing regimen for reliably reproducing the hypothyroid state in mice is well established in the literature [16-20]. PTU administration was initiated 30 minutes after the HOCl subcutaneous injection, and continued for 6 weeks. All agents were prepared fresh daily. Sham-treated animals received injections of 100 μl of saline solution.

### Experimental procedure

At the end of the experiment, animals were killed with an overdose of pentothal sodium (80 mg/kg/intraperitoneally). Serum samples were collected by cardiac puncture from each mouse and stored at −80°C until use. Lungs were removed from each mouse, and a small piece immediately stored for Western blot at -80°C until use, whereas the rest was collected for histopathology, inflated with 400 µl of 10% formalin/PBS, and fixed in formalin for 24 hours. After paraffin embedding, 5-µm sections were cut throughout the whole lung. Five sections, with 1-mm intervals, were stained with Masson Trichrome (MT), and systematically scanned with a light microscope, as previously described [21,22]. A skin biopsy was performed on the back region, involving the skin of the injected area, and stored at −80°C for protein expression or fixed in 10% neutral buffered formalin for histopathologic analysis.

### Determination of Rho, Ras, ERK, and VEGF by Western blot analysis

Lung and skin samples were homogenized in radioimmunoprecipitation assay (RIPA) buffer (25 m*M *Tris/HCl, pH 7.4; 1.0 m*M *EGTA; 1.0 m*M *EDTA) added with 1% of Nonidet P40, 0.5% of phenyl methylsulfonyl fluoride (PMSF), aprotinin, leupeptin, and peptastatin (10 μg/ml each), with a Ultra Turrax (IKA, Staufen, Germany) homogenizer. The lysate was subjected to centrifugation at 15.000 rpm for 15 minutes at 4°C. The supernatant was collected and used for protein determination with the Bio-Rad DC protein assay kit (Bio-Rad, Richmond, CA, USA). Protein samples (30 μg) were denatured in reducing buffer (62 m*M *Tris pH 6.8, 10% glycerol, 2% SDS, 5% β-mercaptoethanol, 0.003% bromophenol blue), and separated by electrophoresis on an SDS (12%) polyacrylamide gel. The separated proteins were transferred on to a PVDF membrane (Amersham, UK), by using the transfer buffer (39 m*M *glycine, 48 m*M *Tris pH 8.3, 20% methanol) at 100 mA for 1 hour. The membranes were blocked with 5% non-fat dry milk (Bio-Rad) in TBS-0.1% Tween for 1 hour at room temperature, washed 3 times for 10 minutes each in TBS-0.1% Tween, and incubated overnight at 4°C with a primary Rho or Ras (Abcam, Cambridge, UK), or ERK, or p-ERK (Cell Signaling, Danvers, MA, USA), or VEGF (Abcam) antibody in TBS-0.1% Tween. After being washed 3 times for 10 minutes each in TBS-0.1% Tween, the membranes were incubated with a peroxidase-conjugated secondary antibody (Pierce, UK) for 1 hour at room temperature. After washing, the membranes were analyzed with the enhanced chemiluminescence system according to the manufacture's protocol (ECL-plus, Amersham, UK). The protein signal was quantified with scanning densitometry by using a bio-image analysis system (Bio-Profil, Milan, Italy). The results from each experimental group were expressed as relative integrated intensity compared with Sham lung or skin tissue measured within the same batch. β-Actin (Cell Signalling) was used on stripped blots to confirm equal protein loading.

### ELISA of serum levels of total T_3 _and T_4 _and TSH

Whole blood was collected from the mice and allowed to clot. The serum was used in ELISA assays to measure total T_3_, total T_4_, and TSH (Mouse Ultrasensitivity Thyroxine, u-T3 ELISA Kit; Mouse Ultrasensitivity Thyroxine, u-T4 ELISA Kit and Mouse ultrasensitive thyroid-stimulating hormone, U-TSH ELISA Kit, MyBiosource, San Diego, CA, USA)

### Histologic and immunohistochemical evaluation of mice

At the end of the experimental phase, lungs and skin were removed from the animals and fixed in 10% buffered formalin, processed for paraffin embedding, sectioned at 5-μm thickness, and subsequently stained with H&E or Masson trichrome, for examination under a light microscope. For immunohistochemistry, paraffin-embedded tissues were sectioned (5 μm), rehydrated, and antigen retrieval was performed by using 0.05 *M *sodium citrate buffer. Tissues were treated with 1% hydrogen peroxide to block endogenous peroxidase activity, and with horse normal serum (Vector Laboratories, Burlingame, CA, USA) to prevent nonspecific staining. A primary antibody against α-SMA (Abcam, Cambridge, UK) was used and kept overnight at 4°C in a humid box. After washing in PBS, a secondary antibody was used (Vector Laboratories), and the location of the reaction was visualized with diaminobenzidine tetra-hydrochloride (Sigma-Aldrich, Milan, Italy). Slides were counterstained with hematoxylin, dehydrated, and mounted with coverslips. As a part of the histologic evaluation, all slides were examined by a pathologist without knowledge of the previous treatment, by using masked slides from ×5 to ×40 magnification with a Leica (Leica Microsystems, Milan, Italy) microscope.

### Measurement of pulmonary MPO activity in mice

Myeloperoxidase activity was determined in lung tissues, after being homogenized in a solution containing 0·5% hexa-decyl-trimethylammonium bromide dissolved in 10 m*m *potassium phosphate buffer (pH 7.0) and then centrifuged for 30 minutes at 20,000 *g *at 4°C. An aliquot of the supernatant was allowed to react with a solution of tetra-methyl-benzidine (1.6 m*m*)//// and 0.1 m*m *H_2_O_2_. The rate of change in absorbance was measured with spectrophotometry at 650 nm. MPO activity was defined as the quantity of enzyme degrading 1 μmol hydrogen peroxide/min at 37° and was expressed in units per 100 mg of tissue.

### Assessment of dermal thickness in mice

Dermal thickness, defined as the thickness of skin from the top of the granular layer to the junction between the dermis and s.c. fat, was examined in histologic samples (Masson trichrome stain) by using the Leica application suite software, as previously described [23,24]. Ten random measurements were taken per section. The results were expressed in micrometers as mean values of dermal thickness for each group. Two investigators in a blinded fashion examined all the sections, independently.

### Assessment of pulmonary fibrosis in mice

The degree of pulmonary fibrosis was evaluated in H&E-stained sections by using the Ashcroft score [25] (0, normal; 1, minimal fibrotic thickening of alveolar walls; 2, moderate thickening of walls without obvious damage to lung architecture; 3, increased fibrosis with definite damage to lung structure and formation of fibrous bands or small fibrous masses; and 4, severe distortion of structure and large fibrous areas. Two pathologists performed all histologic evaluations in a blinded fashion.

### Statistical analysis

All quantitative data are expressed as mean ± SD for each group. Data were compared by using the nonparametric Mann-Whitney test or the Student paired *t *test. When the analysis included more than two groups, one-way analysis of variance was used. *P *values <0.05 were considered significant.

### Results

#### Propylthiouracil administration abated thyroid function

Propylthiouracil, at the dose of 12 mg/kg/s.c./day, determined the inhibition of thyroid function in treated mice compared with the other groups, as shown by the significant decrease in total triiodothyronine (TT_3_) and thyroxine (TT_4_) and the increase in TSH serum levels (Table 1).

**Table 1:** Effects of PTU on serum thyroid hormone levels.

	Sham *(n *= 5)	HOCl (*n *= 10)	HOCl + PTU (*n *= 10 )	
TSH (ng/ml)	1.2 ± 0.4	1.1 ± 0.5	5.4 ± 0.3	*P < 0.001

T_3 _(n*M*)	2.8 ± 0.1	2.9 ± 0.2	0.8 ± 0.5	*P < 0.001

T_4 _(n*M*)	58.8 ± 15.3	60.7 ± 18.1	19.3 ± 2.1	*P < 0.001

#### Propylthiouracil administration prevents dermal fibrosis in HOCl-injected mice

At the end of the experiment, the histologic examination of Masson trichrome-stained skin sections of HOCl-treated mice (HOCl group, *n *= 10), HOCl plus PTU-treated mice (PTU group, *n *= 10), and vehicle alone (Sham group, *n *= 5) demonstrated that HOCl induces dermal fibrosis, as expressed by the increase in dermal thickness, compared with Sham. Moreover, skin samples of HOCl- and PTU-treated mice were strikingly protected from HOCl-induced dermal fibrosis. The simultaneous administration of HOCl and PTU prevented the increase in dermal thickness induced by HOCl. (Figure 1A,B,C,D). In addition, the PTU group had a reduced presence of myofibroblasts, as determined by α-SMA staining when compared with the HOCl group. **(**Figure 2A, B, C, D**)**.

**Figure 1:** **Accumulation of collagen in experimental dermal fibrosis is prevented by propylthiouracil administration**. Dermal thickness was determined by using photomicrographs of Masson-stained sections, by measuring the distance between the epidermal-dermal junction and the dermal-fat junction at 10 randomly selected sites/high-power field (HPF), for 10 HPFs per section. Skin fibrosis was induced in mice by subcutaneous injection of HOCl. The resultant increase in dermal thickness was significantly reduced by subcutaneous injection of propylthiouracil. Representative Masson trichrome-stained sections were examined with light microscopy: (**A) **Normal histology of a representative skin tissue obtained from a Sham mouse; (**B) **Representative histology of skin tissue of HOCl mice; (**C) **Representative histology of skin tissue of HOCl + PTU mouse (original magnification,×10.); (**D) **Dermal thickness in mice from the three experimental groups (Sham group, *n *= 5; HOCl group, *n *= 10; HOCl + PTU group, *n *= 10). Values are expressed as the mean and SD. *P < 0.001 versus Sham #*P *< 0.001 versus HOCl.

**Figure 2:** **Immunostaining for α-SMA (arrows, myofibroblasts nuclei) in cutaneous samples**. Representative tissue sample from: (**A) **Sham animal; (**B) **HOCl mice; (**C) **HOCl + PTU animal (Original magnification, ×40). The arrows show strong diffuse staining of myofibroblasts nuclei (dark brown staining); (**D) **Number of myofibroblasts from the three experimental groups (HOCl + PTU group, *n *= 10; HOCl group, *n *= 10; Sham, *n *= 5). The increase of myofibroblast population in the skin of HOCl mice is prevented by propylthiouracil administration. Values are expressed as the mean and SD. *P < 0.001 versus Sham; #*P *< 0.001 versus HOCl.

#### Propylthiouracil treatment prevents HOCl-induced pulmonary fibrosis

We next investigated whether PTU affects HOCl-induced pulmonary fibrosis. At the end of the experimental procedure, most of the alveolar walls were thickened, the air spaces were collapsed, and collagen deposition in the lungs was markedly present. Semiquantitative assessment by using the Ashcroft score demonstrated that the degree of pulmonary fibrosis in the HOCl (*n *= 10) was significantly higher than in the Sham (*n *= 5) group. In contrast, pulmonary fibrosis was prevented in the PTU (*n *= 10) group (Figure 3A, B, C, D). Myofibroblast differentiation, as determined by α-SMA staining in pulmonary tissues, was less evident in the PTU than in the HOCl mice (Figure 4A, B, C, D).

**Figure 3:** **Preventive effect of propylthiouracil administration upon pulmonary fibrosis development in HOCl-induced murine model of systemic sclerosis**. Representative Masson's trichrome-stained section of lung examined by light microscopy: (**A) **Normal histology of a representative lung tissue from Sham mouse; (**B) **Representative lung section from HOCl mouse; (**C) **Representative lung section from HOCl + PTU mouse (Original magnification, ×10.); (**D) **Semiquantitative analysis of lung tissue graded by using the Ashcroft score, as described in Methods. The degree of pulmonary fibrosis was evaluated in Masson trichrome-stained sections by using the Ashcroft score (the grade of lung fibrosis was scored on a scale of 0 to 8 by using the following criteria: grade 0, normal lung; grade 1 to 2, minimal fibrous thickening of alveolar or bronchiolar wall; grade 3 to 4, moderate thickening of walls without obvious damage to lung architecture; grade 5 to 6, increased fibrosis with definite damage to lung structure; and grade 7 to 8, severe distortion of structure and large fibrous areas. Values are expressed as the mean and SD. *P < 0.001 versus Sham; #*P *< 0.001 versus HOCl. HOCl group (*n *= 10), HOCl + PTU group (*n *= 10), Sham (*n *= 5).

**Figure 4:** **Immunostaining for α-SMA (arrows are illustrative for myofibroblasts nuclei) in pulmonary samples**. Representative tissue sample from: (**A) **Sham animal; (**B) **HOCl mice; (**C) **HOCl + PTU animal (Original magnification, ×40). The arrows show strong diffuse staining of myofibroblasts nuclei (dark brown staining); (**D) **Number of myofibroblasts from the three experimental groups (HOCl + PTU group, *n *= 10; HOCl group, *n *= 10; Sham, *n *= 5). The increase of myofibroblast population in the skin of HOCl mice is prevented by propylthiouracil administration. Values are expressed as the mean and SD. *p < 0.001 versus Sham; #p < 0.001 versus HOCl.

#### High levels of VEGF, p-ERK, RAS, and RHO in cutaneous and pulmonary tissues of HOCl-treated mice are reduced by propylthiouracil treatment

Higher amounts of VEGF, p-ERK, RAS, and RHO proteins were found both in the skin (Figure 5A, B, C, D) and in the lungs (Figure 6A, B, C, D) of HOCl compared with Sham mice, as demonstrated with Western blot analyses. Treatment with PTU significantly reduced the expression of these proteins. No significant difference in the expression of TGF-β (data not shown) was observed in mice exposed to HOCl versus Sham mice or between HOCl and PTU mice.

**Figure 5:** **Effect of propylthiouracil on RAS (A), RHO (B), pERK (C), and VEGF (D) proteins expression in lung tissue samples**. Values in A through D are expressed by the mean and SD relative for each animal group. *P < 0.001 versus Sham; #*P *< 0.001 versus HOCl. HOCl group (*n *= 10), HOCl + PTU group (*n *= 10), Sham (*n *= 5).

**Figure 6:** **Effect of propylthiouracil on RAS (A), RHO (B), pERK (C), VEGF (D) protein expressions in skin tissue samples**. Values in A through D are expressed by the mean and SD relative for each animal group. *P < 0.001 versus Sham; #*P *< 0.001 versus HOCl. HOCl group (*n *= 10), HOCl + PTU group (*n *= 10), Sham (*n *= 5).

#### Myeloperoxidase activity is reduced by PTU administration

To evaluate whether PTU could affect the activity of other peroxidases, than thyroid, pulmonary myeloperoxidase (MPO) activity was tested. This peroxidase, which is itself involved in the production of HOCl and in the oxidative burst, was highly activated in HOCl-treated mice, and significantly reduced by PTU concomitant administration (Figure 7).

**Figure 7:** **Myeloperoxidase (MPO) activation in the lungs is abrogated by propylthiouracil administration**. MPO activity was defined as the quantity of enzyme degrading 1 μ*M *hydrogen peroxide/minute at 37°C and was expressed in units per 100 mg of tissue. *P < 0.001 versus Sham; #*P *< 0.001 versus HOCl. HOCl group (*n *= 10), HOCl + PTU group (*n *= 10), Sham (*n *= 5).

## Discussion

Free radical-mediated oxidative stress has been implicated in the etiopathogenesis of several autoimmune disorders [26]. It seems plausible that in SSc, free radicals contribute to vascular damage and jeopardize the function of the endothelial system, leading to immune system involvement and to fibroblast activation and eventually to tissue fibrosis [27].

Under normal conditions, the antioxidant system of the skin protects cells against oxidative injury and prevents the production of oxidation products, such as 4-hydroxy-2-nonenal or malonaldehyde, which are able to induce protein damage, apoptosis, or release of pro-inflammatory mediators, such as cytokines [28].

Hypochlorous acid (HOCl), the oxygen-reactive species we used to induce systemic sclerosis in our model and the major strong oxidant produced by myeloperoxidase, reacts readily with free amino groups to form *N*-chloramines [29]. HOCl and *N*-chloramines are unstable intermediates that can oxidize thiol groups and cause damage to cells [30]. Plasma thiol concentrations are reduced in patients with SSc compared with controls, suggestive of increased free radical production, and these reduced thiol levels were found in association with white blood cell activation [31]. PTU is a thiol-derived drug, and it could act as an exogenous source of plasma thiols contributing to reduction in the damage mediated by reactive oxygen species. The protective effects of PTU against liver damage, due to its antioxidant activity, have already been reported [32]. Our results show that PTU-treated mice are protected from HOCl-induced damage in the skin (Figure 1A-D). In patients with psoriasis, PTU has been used because of its antioxidant potential and also antiproliferative and immunomodulatory effect [33].

Our study also showed that HOCl-induced pulmonary fibrosis is prevented by PTU treatment (Figure 3A-D). Our findings show that MPO activity is highly activated in HOCl-treated mice, and consequently, PTU administration decreased its activity in the lungs. MPO catalyzes the formation of hypochlorous acid (HOCl), a potent bactericidal agent that is capable of oxidizing and chlorinating a broad spectrum of biomolecular species [34]. Several studies have shown its involvement in oxidative stress and inflammation [35], supporting the central role in the connection between ROS and fibrosis. In cystic fibrosis patients, it has been recently proposed to use thiol-containing molecules as antioxidants, to counteract the MPO system and therefore lung injury [36]. Previous reports showed that propylthiouracil treatment decreases the susceptibility to oxygen radical-induced lung damage in newborn rats exposed to prolonged hyperoxia [37], addressing a role in pulmonary HOCl-induced fibrosis for PTU.

This role may be related to the inhibition of thyroid hormone production, effect on O_2 _metabolism, or its direct antioxidant properties. In an animal model of multiorgan failure after a major burn, PTU-induced hypothyroidism reduced oxidative damage in the hepatic, gastric, and ileal tissues, probably due to hypometabolism, which is associated with decreased production of reactive oxygen metabolites and enhancement of antioxidant mechanisms [38].

In this setting, another study demonstrated that hypothyroidism reduced oxidant stress in kidney and testis tissues, and short-term, high-dose thyroxine administration restored oxidant stress in the same tissues of rats [39].

Moreover, T_3_-induced hyperthyroidism stimulated oxidative damage in rat muscle [40], whereas in hepatic stellate cells (HSCs) isolated from rats treated with thioacetamide (TAA), triiodothyronine (T_3_) and L-thyroxine (T_4_) enhanced activation of HSC and their transdifferentiation in myofibroblasts through activation of Rho. *In vivo*, the administration of T_3 _or T_4 _together with TAA enhances hepatic fibrosis after 3 weeks, compared with the TAA-treated group, accompanied by increased *α*SMA expression in T_3_- and T_4_-treated groups [41], whereas in another study, hepatic fibrosis was significantly reduced in hypothyroid rats, either chemically and surgically induced, as compared with euthyroid controls, and was aggravated in TAA-treated hyperthyroid rats [42].

In SSc patients, hypothyroidism, either clinical or subclinical, has been frequently reported [43], theoretically representing a counterregulatory mechanism against reactive oxygen species damage. In contrast, patients with hyperthyroidism exhibit increased levels of malondialdehyde and myeloperoxidase (MPO) activity in comparison with controls [44]. Treatment with PTU attenuated these increments after 1 month [45]. It has also been shown that PTU can substitute for glutathione as a substrate in glutathione *S*-transferase catalyzed reactions [46].

Our findings imply a central role for ERK-mediated (Figures 5A-D, 6A-D) pathways in the connection between thyroid disease and systemic sclerosis, further supported by the demonstration that the inhibition of Rho and Ras can be associated with amelioration of the fibrotic component present in the disease model based on reactive oxygen species injury. Rho kinase cascade has been shown to be directly involved in the production of collagen by cardiac fibroblasts [47]. A previous report showed that blocking the Ras/MEK/ERK signaling could abolish this fibrotic response *in vitro *[48]. More interestingly, the inhibition of RhoA target protein, Rho-kinase (ROCK), may interrupt signaling pathways known to contribute to pulmonary fibrosis, as already evidenced in bleomycin-induced experimental pulmonary fibrosis [49].

In response to normal tissue injury, fibroblasts migrate into the wound, where they synthesize and remodel new extracellular matrix. The fibroblast responsible for the process of wound healing is called the myofibroblast, which expresses the highly contractile protein α-smooth muscle actin (α-SMA). Abnormal myofibroblast activation is a key feature of fibrotic diseases, including SSc [50]. It was recently demonstrated that blocking ROS with *N*-acetyl cysteine alleviates the elevated contractile and migratory capability of lesional SSc dermal fibroblasts [51] consistent with our results (Figure 2A-D). Postmortem analyses in different stages of SSc lung fibrosis showed that the induction of a large number of smooth muscle α-actin-positive myofibroblasts interstitially characterize, together with overdevelopment of capillary microvessels, the early phase of tissue damage. Our results show that myofibroblast proliferation in the lung is prevented by PTU treatment (Figure 3A-D).

In addition to fibroblast hyperproliferation and collagen hyperproduction, SSc is characterized by vascular abnormalities. One of the predominant growth factors associated with vascular endothelial proliferation, survival, and migration is VEGF [52]. Several groups of investigators have reported that VEGF is upregulated in skin of patients affected by SSc, consistent with our results [53,54]. VEGF could be considered another prooxidative factor when coupled with NOX-4.

An alternative hypothesis is that PTU operates in part at least through a conventional thyroid hormone-mediated mechanism similar the mechanism through ERK, as ascribed to PTU in a rat model of primary pulmonary hypertension [55]. In that model, the thyroid-hormone mechanism was confirmed by thyroidectomy (with no opportunity for antioxidant effect) as well as by PTU. It long has been known that epidemiologic data support a link between both SSc and pulmonary hypertension and thyroid abnormality [56,57]. Clinical trials focusing on patients affected by hyperthyroidism demonstrated that they tend to have elevated pulmonary arterial pressures that are normalized under treatment with thyroid-suppressive therapy [58-60]. These data support the hypothesis that thyroid abnormalities in humans function permissively to facilitate the disease, as demonstrated in the rat model of pulmonary hypertension.

## Conclusions

Although thyroid-function alterations [10-14,43] are frequently reported in SSc patients, our data suggest that PTU exerts an antioxidant effect, consistent with previous reports [31-33,36,37], abrogating the development of cutaneous and pulmonary fibrosis in this animal model of systemic sclerosis. Therefore, further studies will be needed to determine what proportion of the protective PTU effect is related to the inhibition of oxidant stress or oxidant stress-induced myofibroblast differentiation, and could be potentially captured clinically by an antioxidant treatment less complex than PTU, and what proportion of the protective effect is through thyroid hormone mechanisms. This latter would have to be captured clinically by focusing on the intracellular signaling pathway, rather than by blocking thyroid hormones *per se*.

## Abbreviations

AITD: autoimmune thyroid disease; α-SMA: α-smooth muscle actin; EDTA: ethylenediaminetetraacetic acid; ERK: extracellular signal-related kinase; H&E: hematoxylin and eosin; HOCl: hypochlorous acid; HSC: hepatic stellate cells; KH_2_PO_4_: potassium hydrogen phosphate; MEK: MAPK and extracellular signal-related kinase; MPO: myeloperoxidase; NaClO: sodium hypochlorite; NF-κB: nuclear factor kappa-light-chain-enhancer of activated B cells; PBS: phosphate buffered saline; PTU: propylthiouracil; PVDF: polyvinylidene difluoride; Ras: rat sarcoma protein; Rho: Ras homolog gene family; ROCK: Rho-associated protein kinase; ROS: reactive oxygen species; SDS: sodium dodecylsulfate; SSc: systemic sclerosis; TAA: thioacetamide; TBS: tris-buffered saline; TGF-β: transforming growth factor β; TSH: thyroid-stimulating hormone; TT_3_: total triiodothyronine; TT_4_: total thyroxine; VEGF: vascular endothelial growth factor.

## Competing interests

The authors declare that they have no competing interests.

## Authors' contributions

GLB conceived and designed the study, participated in acquisition of data, analysis and interpretation of data, and drafted the manuscript. AB, NI, and GP performed the animal study and histologic and molecular analysis, participated in acquisition of data, analysis and interpretation of data, and revision of the manuscript. DS, CM, MA, and DA contributed to analysis and interpretation of data and the revision of the manuscript. WNR contributed to conception and design of the study and revised the manuscript critically for important intellectual content. GFB, AS, and FS contributed to the design and coordination of the study, analysis and interpretation of data, and revision of the manuscript. All authors read and approved the final manuscript.
